# The Sexual Risk Context among the FEM-PrEP Study Population in Bondo, Kenya and Pretoria, South Africa

**DOI:** 10.1371/journal.pone.0106410

**Published:** 2014-09-17

**Authors:** Jennifer Headley, Ansley Lemons, Amy Corneli, Kawango Agot, Khatija Ahmed, Meng Wang, Jacob Odhiambo, Joseph Skhosana, Jenae Tharaldson, Lut Van Damme, Kathleen MacQueen, for the FEM-PrEP Study Group

**Affiliations:** 1 FHI 360, Durham, North Carolina, United States of America; 2 Impact Research and Development Organization, Kisumu, Kenya; 3 Setshaba Research Center, Soshanguve, South Africa; Rush University, United States of America

## Abstract

**Background:**

Incidence rates in the FEM-PrEP and VOICE trials demonstrate that women from diverse sub-Saharan African communities continue to be at substantial HIV risk.

**Objective:**

To describe and compare the sexual risk context of the study population from two FEM-PrEP trial sites–Bondo, Kenya, and Pretoria, South Africa.

**Methods:**

At baseline we collected information about demographics, sexual behaviors, and partnership beliefs through quantitative questionnaires with all participants (Bondo, n = 720; Pretoria, n = 750). To explore the sexual risk context, we also conducted qualitative, semi-structured interviews with HIV-negative participants randomly selected at several time points (Bondo, n = 111; Pretoria, n = 69).

**Results:**

Demographics, sexual behavior, and partnership beliefs varied significantly between the sites. Bondo participants were generally older, had fewer years of schooling, and were more likely to be employed and married compared to Pretoria participants. Bondo participants were more likely to report multiple partners and not knowing whether their partner had HIV than Pretoria participants. A significantly higher percentage of Bondo participants reported engaging in sex without a condom with their primary and other partners compared to Pretoria participants. We found a borderline association between participants who reported not using condoms in the 4 weeks prior to baseline and lower risk of HIV infection, and no association between having more than one sexual partner at baseline and HIV infection.

**Discussion:**

Despite significantly different demographics, sexual behaviors, and partnership beliefs, many women in the FEM-PrEP trial were at risk of acquiring HIV as demonstrated by the sites’ high HIV incidence. Though gender dynamics differed between the populations, they appear to play a critical role in women’s sexual practices. The findings highlight different ways women from diverse contexts may be at-risk for HIV and the importance of providing HIV prevention options that are both effective and feasible given personal and social circumstances.

## Introduction

Breakthroughs in the field of HIV prevention have identified encouraging approaches to substantially reduce the number of new infections. In recent pre-exposure prophylaxis (PrEP) clinical trials, daily oral emtricitabine (FTC)/tenofovir disoproxil fumarate (TDF) was demonstrated to reduce HIV infection by 75% among serodiscordant couples in Kenya and Uganda [1], by 62% among men and women in Botswana [2], and by 44% among transgender women and men who have sex with men in Peru, Ecuador, South Africa, Brazil, Thailand, and the United States [3]. Among injecting drug users in Thailand, daily oral TDF reduced HIV infection by 49% [4]. In contrast, two trials assessing daily oral FTC/TDF among women in Africa – FEM-PrEP and VOICE – were unable to demonstrate effectiveness for HIV prevention due to low adherence [5], [6].

Women continue to be disproportionally burdened by HIV, particularly in sub-Saharan Africa [7]. The incidence rates from FEM-PrEP and VOICE (5.0 and 5.7 per 100 person years in the placebo arms, respectively) demonstrate that women from diverse communities in sub-Saharan Africa remain at substantial HIV risk [5], [6]. Abstinence, mutual faithfulness, and condom negotiation for HIV prevention continue to be unattainable for many heterosexual women [8]–[17]. Interventions to modify sexual risk factors are not always sufficient, particularly when focused on changing individual behaviors that do not account for structural barriers, the broader social environment, or the gender identities from which sexual behaviors stem [17]–[20]. New prevention technologies, such as PrEP, which may not be reliant on male partner participation, can provide women an option for protection within these contextual constraints and may be effective in altering the course of the epidemic, particularly when paired alongside broader interventions [11], [21]. Additional descriptions of the differences and similarities of sexual behaviors, partnership beliefs, and gender dynamics across different populations can better position future prevention efforts, including PrEP use.

In this paper, we provide a descriptive analysis of sexual behaviors, risk characteristics, and partnership beliefs of the study population from two FEM-PrEP sites – Bondo, Kenya, and Pretoria, South Africa. We describe the trial population at two sites to provide additional descriptions beyond that which is presented in the primary article [5] and to capture and compare the behaviors, partnership beliefs, and contexts that led to the high incidence rates.

For the Bondo site, we recruited from both Bondo and Rarieda (population of 320,092). Bondo and Rarieda are located in the Nyanza Province in western Kenya and are comprised mostly of men and women from the Luo ethnic community. Polygyny, culturally prescribed sex (e.g., having sex during socially sanctioned events such as planting and harvesting or establishing a home) and widow cleansing and inheritance (i.e., the practice of engaging in sex with a male relative of a deceased husband or with a hired man) are customary among the Luo [22], [23]. Having sex without a condom, as expected during widow cleansing, and men’s concurrent partnerships common to the practice of widow inheritance, increase risk for HIV among widows [22]–[24]. Widows have acknowledged a struggle between protecting themselves from HIV and meeting cultural expectations and livelihood needs [25]. Economic necessities, including the localized “sex for fish” trade around Lake Victoria, also impact women’s ability to negotiate safe sex, as residents rely primarily on the fishing industry and subsistence farming [18], [26], [27].

The Pretoria FEM-PrEP site is located in Soshanguve, an urban municipality north of Pretoria (population 311,223) in the Gauteng province. The population includes people from the Sotho, Shangaan, Nguni, and Venda tribes. Throughout South Africa, black South Africans face high unemployment rates, social inequalities, declining marriage rates resulting in an increase in one-person households, and growing migration between rural and urban settings [28], [29]. Women often rely on informal work, transactional or ‘survival’ sex, and other small, informal enterprises [29], [30]. Gender inequality frequently enforces masculine gender norms, whereby multiple partnerships and physical and sexual violence are used to establish power and to control female partners [31]. Furthermore, while gender identities are diverse, the dominant black feminine identity in South Africa, with social and cultural roots and expectations of a ‘good’ woman, generally complies with the dominant masculine identity of strength, sexual success, infidelity, and control over women, often as a way to secure social or material rewards [20], [32]. In these cases, gender dynamics increase women’s risk for HIV, particularly among young women [20], [31].

## Methods

### FEM-PrEP Study Overview

FEM-PrEP was a Phase III, randomized, double-blind, placebo-controlled clinical trial to assess the safety and effectiveness of FTC/TDF in preventing HIV acquisition among women between 18 and 35 years of age at higher risk for HIV in Bondo, Kenya; Pretoria and Bloemfontein, South Africa; and Arusha, Tanzania [5]. Women who had vaginal sex at least once in the past two weeks or who had more than one sexual partner in the past month were eligible to participate. Women reporting these behaviors were presumed to be at risk for HIV given the sites’ high prevalence and generalized epidemics. Qualitative research on adherence, sexual behaviors, and trial experiences was embedded within the clinical trial protocol at the Bondo, Pretoria, and Arusha sites.

Of the 2,120 women who enrolled in FEM-PrEP, 739 were from Bondo and 764 were from Pretoria. The incidence rates from both sites were high –4.7 and 6.0 per 100 person years in the placebo arms, respectively [5]. Details of the FEM-PrEP clinical trial are provided elsewhere [5]. At the time of the trial’s early closure, the Bondo and Pretoria sites were the only ones to have been fully enrolled; the Arusha site had just begun recruitment.

### Data Collection and Sampling

We used quantitative questionnaires administered by interviewers to collect demographic information at screening and information about participants’ sexual behaviors and relationships at enrollment. Questions assessed whether participants had a primary partner or other sexual partners; frequency of vaginal sex with a primary partner in the last 7 days; number of other sexual partners in the last 7 days; frequency of vaginal sex with other sexual partners in the last 7 days; frequency of condom use during vaginal sex with primary and other partners in the last 4 weeks; whether a participant exchanged money or gifts for sex in the last 4 weeks (as an assessment of sex work); and whether a participant’s primary partner, or other sexual partner from the last 4 weeks, was known to be HIV-infected. Only those women who reported having multiple partners were asked if they had exchanged money or gifts for sex in the last 4 weeks. For this analysis, we use the effectiveness population sample from Bondo (n = 720) and Pretoria (n = 750). The effectiveness population includes all participants who were randomized and excludes participants already infected with HIV at enrollment and those whose status was never determined after enrollment due to loss to follow-up, reporting errors, or otherwise missing data.

We also conducted qualitative, semi-structured interviews (SSIs) every three to four months throughout the implementation of the clinical trial. We used a random sample with replacement of 5% of the HIV-negative participants at each time point. The SSIs had two overall purposes: 1) to collect data on adherence and participants’ trial experiences, which were rapidly analyzed and shared without identifiers with local staff so they could respond quickly to any implementation concerns, and 2) to gather supporting data related to the secondary FEM-PrEP objectives on adherence and sexual behavior. A total of 180 participants from Bondo and Pretoria were interviewed (Bondo, n = 111; Pretoria, n = 69). Ten participants were interviewed twice due to sampling. Since the sites initiated at different times and the trial closed early, fewer participants were interviewed in Pretoria. While all interviews explored participants’ study product adherence and acceptability, a subset of participants (Bondo, n = 72; Pretoria, n = 48) were specifically asked to describe the context surrounding their sexual behaviors and relationships, focusing on the reasons for condom use and non-use with their primary and other partners, their knowledge of whether their partner(s) had other sexual relationships, knowledge of their partner’s HIV status, and experiences with transactional sex. As with the quantitative questionnaires, only those women who reported having multiple partners were asked if they had exchanged money or gifts for sex. The SSIs lasted approximately one hour, were conducted in the language chosen by the participant, and were audio-recorded with the participant’s permission. The audio-taped interviews were then simultaneously transcribed and translated from the local language to English. If a participant declined to be recorded (n = 24, 13%), detailed notes were taken and later expanded.

### Ethics Statement

All qualitative and quantitative data collection instruments were approved as part of the FEM-PrEP clinical trial protocol by The Kenyatta National Hospital/University of Nairobi Research and Ethics Committee in Kenya (Bondo), the Medunsa Campus Research Ethics Committee in South Africa (Pretoria), and FHI 360’s Protection of Human Subjects Committee. As part of the enrollment consent process, participants gave their written consent to participate; willingness to participate in the qualitative interview was verbally reconfirmed with each participant before each interview.

### Analysis

For the questionnaire data, we used descriptive statistics to identify the key sexual behavior characteristics and partnership beliefs at each site that are commonly known to place individuals at risk for HIV. We compared these selected sexual behavior characteristics and beliefs for participants at both sites at enrollment using nonparametric Wilcoxon-Mann-Whitney tests for continuous variables and chi-square/Fisher’s exact tests for categorical variables. We then performed logistic regression to assess bivariate associations between demographic factors (i.e., age, being married, living with a sexual partner, and years of education) and selected sexual behaviors (i.e., having more than one sexual partner and having sex without a condom with a primary partner). We also conducted a survival analysis to test if having more than one sexual partner at baseline or having sex without a condom in the four weeks prior to baseline was associated with HIV infection during the trial, using a Cox model stratified on study site and adjusted by age, education, and treatment. All analyses were performed with SAS version 9.3.

For the SSIs, we used applied qualitative thematic analysis to analyze the data [33]. Instead of limiting the analysis to the subset of participants (Bondo, n = 72; Pretoria, n = 48) who were asked specific questions about their sexual behaviors and relationships, we reviewed all SSI transcripts (n = 190, as 10 participants were interviewed twice; total transcripts: Bondo, n = 118; Pretoria, n = 72) for data related to sexual behaviors. While the extent of sexual behavior data varied by transcript, almost all participant interviews (n = 189) contained relevant sexual behavior and sexual context data. Four analysts applied codes in NVivo 9 using a collaboratively created codebook of structural and thematic codes pertaining to sexual behavior. Structural codes were identified based on interview guide questions and thematic codes were added based on the presence of repeated, emerging topics. Codes included discussion of sexual partners (e.g., partner’s characteristics and belief of HIV status), the dynamics of the participants’ sexual relationships and areas of conflict or support related to sexual behavior, and the participants’ own sexual behaviors (e.g., condom use, transactional sex). Fifteen percent of all transcripts, evenly split between the sites and representing the entire duration of the trial, were independently coded by the four analysts who routinely checked inter-coder reliability by assessing code application for each paragraph manually. Any coding discrepancies were discussed and resolved, revising previously coded transcripts and the codebook if necessary. Based on the selected sexual behavior characteristics in the questionnaire data commonly known to place people at risk for HIV, we analyzed coded segments (both structural and thematic) of related text from the SSIs. Two analysts independently created data reduction tables from the coded segments to identify sub-themes, emergent data that were repeated across multiple codes, and frequencies of responses, which were then summarized with illustrative quotes.

## Results

To illustrate FEM-PrEP participants’ sexual risk context, we describe, by site, participants’ baseline demographics (Table 1), sexual behaviors and beliefs of sexual partners’ HIV status at enrollment (Table 2), and demographic factors associated with sexual behaviors (Tables 3 and 4). For each content area, we provide contextual and descriptive information, gathered from the SSIs, to expand on the HIV risk characteristics identified in the quantitative questionnaire findings and provide additional insight into varying gender dynamics. We then compare the sexual behaviors and sexual risk contexts between the two sites and describe the association between selected sexual behaviors and HIV infection.

**Table 1:** Baseline Demographics.

Variable*	Bondo (N = 720)	Pretoria (N = 750)
**Age – yr**		
Mean	26.6	23.2
18–24	279 (38.8)	518 (69.1)
25–29	200 (27.8)	155 (20.7)
30–35	241 (33.5)	77 (10.3)
**Education – yr**		
Mean	8.5	11.4
Median (Range)	8 (0–16)	12 (0–19)
**Marital Status & Co-Habitation**		
Not currently married, not living with partner	183 (25.4)	628 (83.7)
Not currently married, living with partner	8 (1.1)	68 (9.1)
Married, not living with partner	29 (4.0)	11 (1.5)
Married, living with partner	500 (69.4)	43 (5.7)
**Occupation**		
None/Housewife	152 (21.1)	501 (66.8)
Student	16 (2.2)	165 (22.0)
Daily or salaried wage earner	444 (61.7)	84 (11.2)
Other	108 (15.0)	0 (0.0)

*Data presented are n (%) unless specified.

**Table 2:** Participants’ Sexual Behaviors and Knowledge of Sexual Partner’s HIV Status at Enrollment.

Variable*	Bondo (N = 720)	Pretoria (N = 750)	P-Value^11^
Sexual partners^1^			
Primary partner only	407 (56.8)	649 (87.5)	–
More than 1 sexual partner^2^	309 (43.2)	93 (12.5)	<.0001
Had vaginal sex with primary partner without a condom in last 4 weeks^3^	585 (81.9)	478 (64.5)	<.0001
Number of vaginal sex acts with primary partner in last 7 days, median (range)	2 (0–25)	3 (0–21)	<0.001
Had vaginal sex with other sexual partner(s) in last 4 weeks^4^	231 (32.2)	80 (10.8)	<.0001
Number of other sexual partners in last 7 days^5^, median (range)	1 (0–2)	1 (0–10)	0.04
Number of vaginal sex acts with other sexual partner(s) in last 7 days^6^, median (range)	2 (1–12)	2 (1–10)	0.93
Used condoms during vaginal sex with other sexual partner(s) in last 4 weeks^7^			
Always	99 (42.9)	57 (72.2)	
Not Always	132 (57.1)	22 (27.9)	<.0001
Received money/gifts in exchange for sex in last 4 weeks^5^^,^ 8, n	170	53	
% among total population^4^, (%)	(23.6)	(7.1)	<.0001
% among women with more than 1 sexual partner, (%)	(54.7)	(59.6)	0.41
Primary partner has HIV^9^			
No	333 (46.6)	503 (68.1)	<.0001
Yes	16 (2.2)	7 (1.0)	
Does not know	365 (51.1)	229 (31.0)	
Other sexual partner(s), the last 4 weeks, had HIV^5^^,^ 10			
No	44 (14.2)	24 (26.4)	0.01
Yes	1 (0.3)	1 (1.1)	
Does not know	264 (85.4)	66 (72.5)	

*Data presented are n (%) unless specified.

1 Data are missing from four participants in Bondo and eight participants in Pretoria.

2 Defined as a primary partner and at least one other partner, or multiple other partners without a primary partner.

3 Asked only to participants who reported vaginal sex with primary partner in the last 4 weeks.

4 Asked only to participants who reported having other sexual partner(s), though variable was reconstructed with a denominator that also includes those who only reported a primary partner.

5 Asked only to participants who reported having other sexual partner(s).

6 Asked only to participants who reported vaginal sex with other sexual partner(s) in the last 7 days.

7 Asked only to participants who reported vaginal sex with other partner(s) in the last 4 weeks; data are missing from one participant in Pretoria.

8 Four participants from Pretoria declined to answer.

9 Three Pretoria participants declined to answer; data are missing from seven participants in Pretoria and six in Bondo.

10 Two participants from Bondo declined to answer.

11 P value by chi-square, Fisher’s exact, or Wilcoxon-Mann-Whitney test as appropriate.

**Table 3:** Bivariate logistic regression of demographic factors associated with having more than one sexual partner+.

Factor	Bondo (N = 716)		Pretoria (N = 742)	
	OR (95%CI)	P-value	OR (95%CI)	P-value
Age^1^	1.0 (1.0, 1.0)	.61	1.0 (1.0, 1.1)	.13
Married^2^	0.5 (0.4, 0.7)	.0001	0.9 (0.4, 2.1)	.74
Living with primary partner^2^	0.5 (0.3, 0.6)	<.0001	0.8 (0.4, 1.6)	.55
Years of education^1^	1.0 (1.0, 1.1)	.68	0.9 (0.8, 1.0)	.06

+ Versus having a primary partner only. Sample includes only those who reported having a primary partner only or more than one sexual partner.

1 With each increase of a year.

2 Response is “yes” versus “no”.

**Table 4:** Bivariate regression of demographic factors associated with having sex without a condom with a primary partner +.

Factor	Bondo (N = 706)		Pretoria (N = 735)	
	OR (95% CI)	P-value	OR (95% CI)	P-value
Age^1^	1.1 (1.0, 1.1)	.0005	1.1 (1.0, 1.1)	.0013
Married^2^	3.5 (2.3, 5.2)	<.0001	2.3 (1.2, 4.5)	.0179
Living with sexual partner^2^	3.2 (2.2, 4.8)	<.0001	2.1 (1.3, 3.4)	.0022
Years of education^1^	0.9 (0.9, 1.0)	.07	0.9 (0.8, 1.0)	.0074

+ Versus always using a condom during sex in last 4 weeks. Sample includes only those who reported vaginal sex with a primary partner in the last 4 weeks and those who responded to condom use question.

1 With each increase of a year.

2 Response is “yes” versus “no”.

### Participants from Bondo

#### Demographics

The majority of participants (n = 529, 73%) from Bondo were married, although a sizeable minority of participants (n = 183, 25%) were single and not living with a sexual partner (Table 1). Among the SSIs, ten (9%) participants said they were inherited after the death of their husband, 17 (15%) others reported being in a polygamous relationship, and two (2%) additional participants reported that their husband, while not polygamous, inherited another woman. The majority of participants were 25 years of age or older (n = 441, 61%), the median years of schooling was 8 years, and most (n = 444, 62%) reported having an occupation where they earned a daily wage or salary (Table 1).

#### Sexual partners

Almost all participants (n = 714, 99%) reported having a primary partner in the questionnaire. Most participants reported having *only* a primary partner (n = 407, 57%) while many others (n = 309, 43%) reported having more than one sexual partner. Among women who reported having other, non-primary sexual partner(s), the median number of partners in the last 7 days was one (Table 2). Participants who lived with a primary partner or who were married were less likely to have multiple partners than those who lived separately from their primary partner or who were not married (Table 3).

In the SSIs, participants described a range of relationships, including husbands, casual partners, boyfriends, and inheritors. Of the 103 participants who described the number of their sexual partners in response to a direct question on the interview guide or in reference to a related question, 51 discussed currently or previously having sexual partners in addition to their primary partner. Some participants elaborated that these concurrent partners were generally casual, and in several cases, living in another area. Some participants also explained that they had other sexual partners because their primary partner was often absent (e.g., migrant work) or because they believed their primary partner was unfaithful:

*“I was having sex with these people because my husband was outside [away from home] and I also had these other people nearby at home” (35-year-old woman in polygamous marriage, whose husband works in Kisumu)*

Among the 309 participants who reported having multiple partners in the quantitative questionnaire, 55% (n = 170) reported exchanging sex for money or gifts. During the SSIs, 18 participants described instances of transactional sex. Most described receiving monetary compensation (n = 16) or a direct exchange of non-monetary assistance such as food, clothes, and goods, including fish (n = 13). One participant explains:

*“Based on the kind of work that he does for me (provides fish), that is why I want to keep him close to me because of the way they are. I mean that if you are not close to him, you can end up that your boat goes to the lake but you do not get any fish; therefore if you keep him close he will work for you as you want and you will get the fish and sell them…. Fishermen are difficult, having sex with him is the only way [I] can keep him close and this is without the husband’s knowledge… you are the one who knows since I am the one who takes the fish.” (25-year-old married woman)*

#### Condom use

Reports of sex without a condom were common. A majority of participants (n = 585, 82%) reported that they had vaginal sex with their primary partner in the last 4 weeks without using a condom (Table 2). Several factors were significantly associated with this behavior including being older, being married, and living with their primary partner (Table 4). Among participants reporting having sex with another partner in the last 4 weeks, 57% (n = 132) reported that they did not always use a condom with one or more of those partners (Table 2).

In the SSIs, 31 participants described the context surrounding condom use with their partner. A few said they did not use condoms because they believed in their partner’s fidelity. On the other hand, believing that partners were or may have been unfaithful did not necessarily result in condom use either; a few women described not using condoms with partners with whom they were uncertain about their “movements” (i.e., sexual behaviors outside of their relationships). A few participants also described how the perception of being a “wife” or “girlfriend” in a committed relationship influenced their inability to use a condom:

*“He said that as someone who is his wife he cannot use [a condom] with me, a condom he can use with someone who is from outside but not in his own house.” (31-year-old married woman)*

More often, participants explained that factors related to power and gender dynamics, specifically the refusal by the male partner to use a condom, prevented condom use:

*“The person I had could at times accept to use it [a condom] or at times he refused. And you know I could not force him to use it because he would tell me what he says is final.” (31-year-old married woman)*

#### Knowledge of Sexual Partners’ HIV Status

About half of participants (n = 365, 51%) reported not knowing if their primary partner had HIV or reported that their partner did not have HIV (n = 333, 47%); however, very few (n = 16, 2%) reported *knowing* that their primary partner had HIV. Similarly, the majority of participants (n = 264, 85%) with multiple partners reported not knowing if their other partners had HIV, while only one participant reported *knowing* that another partner had HIV (Table 2).

In the SSIs, 73 participants discussed their primary partner’s HIV status. Participants (n = 18) who did not know their partner’s status most often described their partner’s refusal to be tested for HIV. As one participant explained:

*“…he is the type of person who does not accept to be tested so you know … he may have HIV and I don’t have … I still don’t know his status until the day he will go for the test is when I will know whether he is positive or negative. But he has refused to go for the test.” (27-year-old married woman)*

A few participants described that a partner’s mobility or living apart from one another was a barrier to knowing his HIV status. Others described that their partners would tell them they are HIV-negative, though without providing, or necessarily having, any evidence:

*“…he just comes for one or two or three days then goes back to Eldoret and I do ask him if he still goes for test to know his HIV status and he accepts [gets tested]. You know someone can just accept [agree that] he goes for a test because there is no proof so I cannot know the truth about that.” (34-year-old married woman)*

Seventeen participants discussed the HIV status of their other sexual partners in the SSIs and almost all (n = 14) said that they did not know. About half of these participants added that they used condoms with these partners for protection because their status was unknown.

### Participants from Pretoria

#### Demographics

A large majority of participants from Pretoria were not married (n = 696, 93%) and most were between 18 and 24 years of age (n = 518, 69%). The median years of schooling was 12 years, and a large majority (n = 666, 89%) reported no income by either not having an occupation or being a student (Table 1).

#### Sexual Partners

Almost all participants (n = 742, 99%) reported having a primary partner, most of whom reported having *only* a primary partner (n = 649, 88%) (Table 2). In the SSIs, 69 participants discussed their primary partners and most often they were described as boyfriends from whom they lived apart:

*“I have one boyfriend and he stays in Sunnyside, but then during weekends he is at home here in Soshanguve.” (19-year-old unmarried woman)*

Thirteen percent (n = 93) of participants reported having more than one sexual partner; the number of other, non-primary partner(s) that participants had sex with in the last 7 days ranged from 0 to 10 with a median of one (Table 2). In the SSIs, participants would at times refer to these partners as casual or unofficial sex partners (e.g., “makhwapeni” or “roll-ons”). Among the 93 participants who reported having multiple partners, 60% (n = 53) reported in the questionnaire exchanging sex for money or gifts, and four participants (4%) declined to answer. None of the participants in the SSIs, however, described engaging in transactional sex.

#### Condom use

Reports of having sex with a primary partner without a condom were common (n = 478, 65%), while fewer women (n = 22, 28%) reported having sex without a condom with other sexual partners (Table 2). Factors significantly associated with sex with a primary partner without a condom included being older, being married, and living with a primary partner. With each additional year of schooling, participants were significantly less likely to report sex with a primary partner without a condom (Table 4).

In the SSIs, 36 participants described the context surrounding condom use with their partner. Some (n = 11) expressed confidence that their primary partner was faithful and therefore they trusted him and saw no reason to use condoms (either at the time of the SSI or previously):

*“He has been with me for a long time, we trust each other. There is no need to use a condom.” (23-year-old unmarried woman)*

Along with trust, some participants accepted having sex without a condom because they did not perceive themselves to be at risk for HIV, they knew their partner’s HIV status, or their partner resisted condom use. A few participants described that feeling comfortable at times with their partner led to inconsistent condom use:

*“So, like sometimes you feel like ehh…let us not use it [condoms], but more often you use it and then maybe sometime I don’t use it because I feel relaxed, maybe he is not doing anything [i.e., having sex with other partners] and I am not doing anything.” (20-year-old unmarried woman)*

#### Knowledge of Sexual Partners’ HIV Status

Most participants (n = 503, 68%) said that their primary partner did not have HIV, 31% (n = 229) reported that they did not know the partner’s status and very few (n = 7, 1%) reported *knowing* that the partner had HIV. In contrast, a majority of participants (n = 66, 73%) reported not knowing if their other sexual partners had HIV and only one participant (1%) reported *knowing* another partner had HIV (Table 2).

In the SSIs, 43 participants discussed their primary partner’s HIV status. Some women described knowing their partner’s HIV status through joint testing:

*“We once went and got tested when we started going out. […] We got tested for the first time in 2007 and sometime, if I remember very well, last year here.” (34-year-old unmarried woman)*

Among those who did not know their primary partners’ HIV status, partner refusal to get tested was one of the most-cited reasons, along with his assertion that her HIV testing could serve as a proxy of his negative status:

*“He is hiding behind my status saying that just because I know mine it means he does not have it [HIV] too. But I do tell him that I don’t always know where he is and with who but he insists he does not have it. So, you cannot force anyone to get tested if he does not want ‘cause he will think you don’t trust him. So, I just leave it like that.” (19-year-old unmarried woman)*

### Comparative Findings

Demographic characteristics, as reported in the questionnaire, varied significantly between the Bondo and Pretoria sites (p<0.001). Participants in Bondo were generally older, had fewer years of schooling, and were more likely to be employed and married. Almost all of the sexual behaviors and partnership beliefs also varied significantly between the two sites (Table 2), with participants from Bondo being more likely to report multiple partners and not knowing whether their partner had HIV. Among the total population, participants from Bondo were significantly more likely to have engaged in transactional sex. However, when assessing transactional sex among only those participants who reported more than one sexual partner, there was no significant difference between the two sites. A significantly higher percentage of participants from Bondo reported engaging in sex with their primary partner without a condom, while a significantly lower percentage reported condom use with their other partners. In both sites, however, being older, being married, and living with a primary partner were all significantly associated with having sex with a primary partner without a condom.

### Sexual behaviors and HIV infection

We did not find a significant association between reporting having more than one sexual partner at baseline and HIV infection [hazard ratio (HR) = 1.25, p = 0.464]. However, women who reported not using a condom in the 4 weeks prior to baseline had a borderline significantly lower risk of HIV infection during the trial compared to women who did report using condoms in the 4 weeks prior to baseline (HR = 0.59, p = 0.052).

## Discussion

FEM-PrEP enrolled women into a clinical trial cohort from two culturally and geographically distinct communities, and high rates of HIV incidence were observed in both sites. In this manuscript, we described the context surrounding such high incidence rates and compared the similarities and differences between the two sites. Despite similarly high HIV incidence rates, sexual risk characteristics, behaviors, and partnership beliefs often varied between participants from the two sites, as we observed differences in marital status, having multiple partners, transactional sex, and knowing whether or not their partners had HIV. However, reports of sex without a condom with their primary partner were common in both sites. SSI data illustrated the on-going barriers to consistent condom use that women from both communities faced, whether due to partner resistance, trusting a partner, or not seeing a reason to use one. These data suggest that condoms were not a viable option for many women, despite more than a decade of condom use campaigns and advocacy. Limited condom use in areas of high HIV prevalence and the barriers to their use, as seen among FEM-PrEP participants, have been frequently reported in the literature [36]–[38]. We also found a borderline significant association between reported sex without a condom at baseline and lower risk of HIV infection after adjusting for age, education, and treatment group. However, this association is likely confounded by other, unmeasured variables (e.g., partners’ HIV status) or changes in condom use patterns during follow-up.

While reports of transactional sex among the total site populations varied between the two sites, when looking specifically at women with other sex partners, the two sites held similar percentages (55% in Bondo, 60% in Pretoria). However, the total number of sexual partners in the previous 7 days reported by participants was low, particularly in Bondo. Moreover, in the SSIs, Bondo participants described money and goods received from boyfriends and casual partners rather than clients. Together, these findings suggest that in Bondo some participants may not have been engaging in professional sex work, but in transactional sex as a way to supplement other sources of income or to obtain goods they needed to conduct their business, such as in the fish trade.

Self-reported data on sexual behaviors are always subjected to recall and social desirability bias. Participants may not have recalled their experiences accurately or they may have over-reported condom use or under-reported the number of sexual partners to comply with cultural norms regarding sexuality or messages they received during the study’s risk reduction counseling. While we implemented strategies to reduce recall and social desirability bias (e.g., conducting the qualitative interview prior to counseling, having separate staff conduct risk reduction counseling from those who interviewed participants), these biases may still exist. We also described the quantitative data from enrollment, while the SSI data was collected at later follow-up visits. Though sexual behaviors can change over time, the questionnaire and SSI findings were comparable.

In many ways, the two trial communities are reflective of the HIV epidemic patterns of their country and region. Throughout South Africa, black African women aged 20–34, and men and women aged 15–49 years old who live together but who are not married, comprise the two key populations identified as most-at-risk with respective HIV prevalences of 32% and 31% [34]. While in Kenya, the Nyanza Province has the highest HIV prevalence at 15% of any region in Kenya. Women aged 25–34 years old within Nyanza Province have the highest prevalence (23%) of any age group and any region [35]. In Kenya, HIV prevalence was also highest amongst persons who had been widowed aged 15–64 years old [35]. Furthermore, in both South Africa and Kenya, women in most age groups are disproportionately affected by HIV compared to men [34], [35]. The high rates of HIV incidence observed in Bondo and Pretoria during FEM-PrEP, placed within the overall context of the HIV epidemic in these respective regions, demonstrate the substantial risk of acquiring HIV that many FEM-PrEP participants faced.

In summary, these data demonstrate that despite significantly different demographics, sexual behaviors, and partnership beliefs between the two study sites, HIV incidence rates were similarly high and therefore many of these women were at risk of HIV exposure. Condoms are a viable choice for some women, but not for most of the women in the two sites, particularly those who are older, married, and living with a primary partner. While not a study on gender, our findings are suggestive of a number of ways gender dynamics can influence a woman’s sexual practices: a dependence on a male partner to agree to and participate in condom use and HIV testing, reduced sexual agency and condom use as a relationship progresses to marriage or living with their partner, multiple sexual partnerships influenced by a primary partner’s proximity, and a potential protective effect in condom use offered by schooling. Our findings illustrate how gender dynamics and inequities may affect sexual practices similarly and dissimilarly across diverse contexts, supporting other social science research that highlights gender dynamics as a critical driver of HIV [20], [39]–[42]. Ultimately, new HIV prevention options are needed to support women in choosing methods that are both effective and feasible given their particular personal and social circumstances. PrEP, known to be effective in preventing HIV, is another option that may work for some women.
